# Properties of Doublecortin-(DCX)-Expressing Cells in the Piriform Cortex Compared to the Neurogenic Dentate Gyrus of Adult Mice

**DOI:** 10.1371/journal.pone.0025760

**Published:** 2011-10-13

**Authors:** Friederike Klempin, Golo Kronenberg, Giselle Cheung, Helmut Kettenmann, Gerd Kempermann

**Affiliations:** 1 ISCRM, Institute for Stem Cell and Regenerative Medicine, University of Washington, Seattle, Washington, United States of America; 2 Department of Neurology and Center for Stroke Research Berlin, Charité University Medicine Berlin, Berlin, Germany; 3 Max-Delbrück-Center for Molecular Medicine (MDC) Berlin-Buch, Berlin-Buch, Germany; 4 Center for Integrative Physiology, School of Biomedical Sciences, University of Edinburgh, Edinburgh, United Kingdom; 5 CRTD –Center for Regenerative Therapies Dresden, Technische Universität Dresden, Dresden, Germany; University of South Florida, United States of America

## Abstract

The piriform cortex receives input from the olfactory bulb and (via the entorhinal cortex) sends efferents to the hippocampus, thereby connecting the two canonical neurogenic regions of the adult rodent brain. Doublecortin (DCX) is a cytoskeleton-associated protein that is expressed transiently in the course of adult neurogenesis. Interestingly, the adult piriform cortex, which is usually considered non-neurogenic (even though some reports exist that state otherwise), also contains an abundant population of DCX-positive cells. We asked how similar these cells would be to DCX-positive cells in the course of adult hippocampal neurogenesis. Using BAC-generated transgenic mice that express GFP under the DCX promoter, we studied DCX-expression and electrophysiological properties of DCX-positive cells in the mouse piriform cortex in comparison with the dentate gyrus. While one class of cells in the piriform cortex indeed showed features similar to newly generated immature granule neurons, the majority of DCX cells in the piriform cortex was mature and revealed large Na+ currents and multiple action potentials. Furthermore, when proliferative activity was assessed, we found that all DCX-expressing cells in the piriform cortex were strictly postmitotic, suggesting that no DCX-positive “neuroblasts” exist here as they do in the dentate gyrus. We conclude that DCX in the piriform cortex marks a unique population of postmitotic neurons with a subpopulation that retains immature characteristics associated with synaptic plasticity. DCX is thus, per se, no marker of neurogenesis but might be associated more broadly with plasticity.

## Introduction

Newly born granule cells in the adult dentate gyrus (DG) express a series of transient markers, such as the microtubule associated protein DCX, the polysialylated neural cell adhesion molecule PSA-NCAM, Tis21, and Calretinin [1], [2], [3], [4], [5]. Quite generally, the expression of doublecortin has been linked to structural plasticity and morphological changes associated with migration, axonal guidance and dendrite sprouting [6], [7], [8], [9], [10]. During development, DCX is necessary for lamination of the hippocampus [11]. In adult hippocampal neurogenesis DCX marks the period between the committed progenitor cell stages (type-2b/3) and the early postmitotic maturation stage and is absent from the radial-glia-like stem cells (type-1), the non-committed progenitor cells (type-2a) and the mature neurons. DCX-positive (DCX+) cells in the dentate gyrus receive synaptic GABAergic input and migrate into the inner third of the granule cell layer [4], [12], [13], [14]. DCX+ cells are also found in the neurogenic subventricular zone (SVZ) of the lateral ventricle, where they mark the migratory A cells [1]. The function of DCX in adult hippocampal neurogenesis is not known, but in many instances DCX-expression is used as surrogate marker of neurogenesis.

However, in the adult rodent brain, DCX expression is not limited to the hippocampus and the subventricular zone/olfactory bulb. DCX-positive cells are found, for example, in the striatum [15], [16], migrating in and below the corpus callosum [17], [18], or in the piriform cortex [19], [20]. Throughout the cortical parenchyma one finds satellite cells positive for proteoglycan NG2, often co-expressing DCX. Yet, little is known about the properties of DCX+ cells outside the “canonical” neurogenic regions in the hippocampal dentate gyrus and the subventricular zone/olfactory bulb system.

As discussed in detail elsewhere, we define the neurogenic regions as characterized by the presence of neural precursor cells, able to generate neurons, and a permissive microenvironment, the niche, together forming one functional unit [21], [22]. By this standard, the adult brain of rodents and primates has two neurogenic regions, while, for example, zebrafish have many more [23]. Neither the term, nor the concept does preclude that new neurons might be found elsewhere, either as exceptional physiological event or in cases of pathology. With the exception of a report on reactive neurogenesis in cortical layer I after stroke [24], such cases of neurogenesis in non-neurogenic regions [16], [25], [26] all imply a relationship of that process to the neurogenic zone of the SVZ.

Here, we characterized DCX-expressing cells in the adult piriform cortex and investigated the significance of a transient immature “neuronal” marker in a region that by this standard is regarded as non-neurogenic (see also [20]). Based on morphological criteria and anatomical location the three-layered structure of the piriform cortex comprises semilunar and pyramidal principal cells in layer II (grouped into semilunar-pyramidal neurons), deep/large pyramidal neurons in layer III and a variety of interneurons that control different parts of the neuronal network with a subpopulation characterized as neurogliaform cells [19], [27], [28]. Layer II contains a high density of principal cells that receive afferent projections from the olfactory bulb (Fig. 1), where a large amount of structural plasticity including adult neurogenesis is found. The piriform cortex is part of the parahippocampal cortices and is often recruited in temporal lobe epilepsy [29]. Such recruitment is associated with a strong increase in cell proliferation [30].

**Figure 1:** Localization and wiring of the piriform cortex. (**A**) Position of the piriform cortex in the circuitry of the olfactory system. The schematic drawing is based on information from [53]. (B) Principal network of the piriform cortex.

One report has claimed the migration of newly generated neurons to the piriform cortex from the ventricular subependyma [31] and two studies indicated inducible neurogenesis in the piriform cortex in a model of vascular dementia [32] or after olfactory bulbectomy [33]. A few other similar claims have been made [34], [35], [36]. To date no report providing the same kind and level of evidence that is available for the hippocampus and olfactory bulb has been published (i.e. the demonstration of developmental stages, functional maturation, etc.). In any case, however, it is intriguing that in the olfactory pathway from the olfactory bulb to the hippocampus, we have two neurogenic zones with abundant DCX expression and one intermediate relay station in the piriform cortex, which also harbors DCX-positive cells.

The transgenic expression of green fluorescent protein (GFP) represents a very powerful tool to visualize cell types, in which a specific promoter is active [37]. We have previously used this approach to characterize nestin-expressing cells in the dentate gyrus [12], [38]. Here, we made use of DCX-GFP transgenic mice to characterize DCX expression in cells of the non-neurogenic piriform cortex compared to the neurogenic niche in the adult hippocampus. We used the DCX-reporter mouse from the Genesat project [39]. Other transgenic DCX reporters have been described [40], [41].

We show that in the piriform cortex, DCX cells are strictly postmitotic with a large subset displaying action potentials. In addition, a small group of postmitotic cells had similar features to newly born neurons of the DG, presumably associated with particular plasticity. Due to synaptic connections of piriform cortex neurons with olfactory bulb interneurons, these cells may be able to adapt to fast environmental changes, and constitute a unique population in adult cortical brain regions.

## Materials and Methods

### Animals and treatment

The BAC transgenic mouse line expressing enhanced green fluorescent protein (eGFP) under the DCX promoter was developed within the Gene Expression Nervous System Atlas (GENSAT) BAC Transgenic Project and obtained from Rockefeller University (http://www.gensat.org). The DCX-GFP mice were established on a FVB/N background. Their generation has been described in detail elsewhere [39].

Animals were six to eight weeks old and weighed 18–22 g at the beginning of the experiments. The mice were held five per cage under standard laboratory housing conditions with a light/dark cycle of 12 hours each and free access to food and water. All experiments were performed according to national and institutional guidelines and were approved by the appropriate authority, Landesamt für Arbeitsschutz, Gesundheitsschutz und technische Sicherheit (LAGetSi) of the State of Berlin, approval numbers G 0312/00 and G 0093/05. Thymidine analog BrdU (5-Bromo-2′-deoxyuridine; SIGMA-Aldrich, Germany) was administered intraperitoneally at a concentration of 50 mg/kg body weight. Animals were killed 24 hours or three days after a single BrdU injection. One group of animals received a three-day series of single BrdU injections and was killed two weeks following the last BrdU injection.

### Immunohistochemistry and imaging

Mice were deeply anesthetized with ketamine and perfused transcardially with 0.9% sodium chloride followed by 4% paraformaldehyde (PFA) in 0.1 M phosphate buffer. Brains were postfixed in 4% PFA at 4°C over night, and transferred into 30% sucrose for dehydration. Brains were cut on a sliding microtome (Leica, Bensheim, Germany) in the coronal plane into 40 µm thick sections and cryoprotected. Sections were stained free floating with all antibodies diluted in Tris-buffered saline containing 3% donkey serum and 0.1% Triton X-100. For BrdU staining, DNA was denatured in 2N HCl for 30 minutes at 37°C.

Primary antibodies were applied in the following concentrations: anti-BrdU (rat, 1∶500; Harlan Seralab, Indianapolis, IN), anti-GFP (green fluorescent protein, rabbit, 1∶400; Abcam, Cambridge, UK), anti-GFP (goat, 1∶1000; Acris Antibodies, DPC Biermann, Germany), anti-S100β (rabbit, 1∶2500; Swant, Belinzona, Switzerland), anti-NeuN (mouse, 1∶100; Chemicon, Temecula, CA), anti-DCX (goat, 1∶200; Santa Cruz Biotechnologies, Santa Cruz, CA), anti-Calretinin (rabbit, 1∶250; Swant, Switzerland), anti-GFAP (guinea pig, 1∶1000; Advanced ImmunoChemistry), anti-NG2 (rabbit, 1∶200; Chemicon, Temecula, CA), and anti-Parvalbumin (goat, 1∶500; Swant, Switzerland).

Immunohistochemistry followed the peroxidase method with biotinylated secondary antibodies (all: 1∶500; Jackson ImmunoResearch Laboratories, West Grove, PA), ABC Elite reagent (Vector Laboratories, Burlingame, CA) and diaminobenzidine (DAB; Sigma) as chromogen. For immunofluorescence FITC-, RhodRedX- or Cy5-conjugated secondary antibodies were all used at a concentration of 1∶250. Fluorescent sections were coverslipped in polyvinyl alcohol with diazabicyclooctane (DABCO) as anti-fading agent.

Confocal microscopy was performed using a spectral confocal microscope (TCS SP2; Leica, Nussloch, Germany). Appropriate gain and black level settings were determined on control tissues stained with secondary antibodies alone. All images were taken in sequential scanning mode and further processed in Adobe Photoshop 7.0 for Macintosh.

### Acute brain slice preparation

Acute brain slices of n = 9 adult transgenic DCX-GFP mice were prepared as described previously [12], [13]. Briefly, mice were decapitated, the brains were removed, washed, and placed in bicarbonate-buffer salt solution at 4°C. The standard bath solution contained in mM: NaCl, 134; KCl 2.5; MgCl_2_, 1.3; CaCl_2_, 2; K_2_HPO_4_, 1.25; NaHCO_3_, 26 and 10 D-Glucose, equilibrated with 95% O_2_ and 5% CO_2_, pH 7.4. The brains were cut into 150 µm thick coronal sections with a Vibratome (Microm HM650V, Walldorf, Germany). Brain slices were immediately transferred with a pipette to a recording chamber installed on the stage of an upright microscope (Axiovert FS, Zeiss, Oberkochen, Germany).

### Electrophysiology

GFP+ cells located in the subgranular zone of the adult DG and the piriform cortex were identified by fluorescence microscopy with excitation at 488 nm generated by a monochromator (Polychrome IV, Till Photonics, Graefelfing, Germany). The emitted light at 530±10 nm was visualized with standard fluorescence optics and captured with a CCD camera QuantiCam (Phase, Luebeck, Germany). Whole cell patch-clamp recordings were performed using an EPC 9 patch-clamp amplifier in combination with the TIDA software (HEKA, Lambrecht, Germany). Patch pipettes were pulled from borosilicate capillaries (inner and outer diameter 0.87 and 1.5 mm; Hilgenberg, Malsfeld, Germany) using a P-2000 laser-based pipette puller (Sutter Instrument, Novato, California). The pipette solution contained in mM: 130 KCl, 2 MgCl2, 0.5 CaCl2, 5 EGTA, and 10 HEPES, pH 7.3. To confirm intracellular access, 10 µg/ml Alexa Fluor 594 (Invitrogen, Karlsruhe, Germany) was always added to the pipette solution. Cells filled with Alexa Fluor 594 were detected at an excitation and emission wavelength of 589 and 616±4 nm, respectively. The open resistance of the patch pipettes ranged from 5 to 8 MΩ. All experiments were performed at room temperature (21 to 25°C).

### Statistical analysis

All numerical analyses were performed using Statview 5.0.1 for Macintosh. ANOVA was followed by Fisher's post hoc test, where appropriate. All values are given as mean ± standard error of the mean (SEM). *P*-values of <0.05 were considered statistically significant.

## Results

### DCX-GFP expression reflects native DCX expression in the adult brain

In the adult mouse brain DCX-GFP was strongly expressed in the hippocampal dentate gyrus (Fig. 2A) and the SVZ of the lateral ventricle (Fig. 2B). However, GFP expressing cells were not confined to the neurogenic regions only, but were, for example, also detected in the stratum oriens of the hippocampal CA1 region (Fig. 2C), and in layers II and III of the non-neurogenic piriform cortex (Fig. 2D). Having previously investigated DCX-positive cells in CA1 [42] we now turned to the corresponding cells in the piriform cortex.

**Figure 2:** DCX-GFP expression and its distribution in the adult brain. (**A–B**) GFP (in green) is expressed abundantly in progenitor cells of the adult dentate gyrus (A) and subventricular zone (B) that also incorporated BrdU (red). (**C–D**) GFP is not only confined to neurogenic regions but also observed in the stratum oriens of the CA1 field of the hippocampal formation (C) where also proliferating cells could be detected (BrdU in red), and the adult piriform cortex (D). Notably, here no proliferation of GFP+ cells was observed at either time.

Figure 2 also shows that GFP+ cells of the DG, SVZ and stratum oriens had incorporated the thymidine analog BrdU. This was not the case for the piriform cortex.

Images in Figure 3 show DCX-GFP vs. DCX peptide expression in the hippocampal DG. Transgenic DCX-GFP mice (Fig. 3A) displayed relatively faint GFP expression in dendritic trees branching into the molecular layer as compared to direct staining against DCX (Fig. 3B). Short basal immature dendrites are typical of newly generated granule cells [14], [43], [44]. GFP expression was detected in the nucleus and soma of cells located in the subgranular zone (SGZ), inner granule cell layer (GCL), and fainter in some hilar interneurons (Fig. 3C). DCX-GFP expression was retained in some migrating intermediate progenitor cells (type-3). For quantitative results, 181 GFP-expressing cells out of 200 cells analyzed (n = 4) showed overlap with the DCX-protein in the SGZ and vice versa 178 DCX+ cells out of 200 cells analyzed showed GFP-expression (Fig. 3C1).

**Figure 3:** Transgenic DCX-GFP expression in comparison with DCX-antigen labeling in the adult mouse DG. (**A–B**) DAB immunoreactivity reveals strong staining in nucleus, soma and proximal processes of GFP+ cells (A) in the granule cell layer (GCL) and weak expression in dendritic trees branching into the molecular layer (ML) relative to DCX-protein (B). A few cells had migrated into the inner GCL (arrow in A); Scale bar 40 µm. (**C**) Confocal images of GFP expression reveals strong staining of progenitor cells in the DG (arrows), and some weak labeling in hilar interneurons (asterisk). (**C1**) GFP and DCX-antigen labeling matches to approximately 90%, but GFP is down regulated in more mature neurons although DCX-protein is still present (arrowhead). Scale bar 100 µm.

### DCX-GFP expression in the adult dentate gyrus as indicator for neurogenesis

Next, we characterized the appearance of GFP+ cells in the course of adult neurogenesis according to our previously developed classification [45]. GFP is transiently expressed during type-2b and type-3 cell stages of neuronal development (as detected with anti-DCX-antibodies, Fig. 3C1) as well as in immature postmitotic neurons (here overlapping with the expression of Calretinin, CR) [3]). Yet, it is absent from mature granule cells and glia-like type-1 stem cells (as identified with GFAP). Quantitatively 72 cells out of 200 GFP+ cells analyzed in the SGZ of transgenic mice (equal to 36%, n = 4) displayed colabeling with the transient and early postmitotic marker CR (Fig. 4A). Conversely, 70% of CR+ cells expressed GFP (140 CR+ cells out of 200 cells analyzed; n = 4). Only 14% of GFP+ cells coexpressed the neuronal marker NeuN (28 out of 200 cells; n = 4; Fig. 4B). We have previously reported that DCX expression occurs primarily at later stages of granule cell development (70% of type-3 cells and early postmitotic neurons express DCX as detected by antigen-labeling) [14]. Transgenic DCX-GFP expression in the hippocampus seems to visualize primarily the actively dividing precursor cell stages type-2a and type-2b and compared to the presence of endogenous DCX protein shows somewhat reduced overlap with postmitotic neuronal markers CR and NeuN.

**Figure 4:** Phenotypes of DCX-GFP-expressing cells in the adult DG. (**A–B**) In the course of adult neurogenesis some of GFP+ cells co-express the early transient postmitotic marker Calretinin (CR, in A) and the lasting postmitotic neuronal marker NeuN (B), indicating that DCX is present in immature neurons. DCX-GFP-positive cells with rounded or flattened nuclear morphology, negative for the other markers represent the precursor cells at the type-2b and type-3 stage (compare [14]). DCX-GFP is absent from the radial glia-like neural stem cells (type-1 cells) and astrocytes as detected with GFAP (C) and S100β (D). S100β-positive cells represent postmitotic astrocytes, some of which are produced in the course of adult neurogenesis. (**E**) A few GFP+ cells express NG2 near to the subgranular zone (SGZ). (**F**) Some of the fainter GFP+ cells in the hilus are colabeled with the interneuron marker Parvalbumin. GCL, granule cell layer; BrdU in red; Scale bar, 120 µm.

Neither native DCX nor transgenic DCX-GFP were expressed in GFAP-expressing type-1 cells (Fig. 4C; [46]). Further phenotypic analysis of GFP+ cells revealed no overlap with the astrocytic marker S100β (Fig. 4D). Some of the fainter GFP+ cells in the hilus and SGZ showed expression of the proteoglycan NG2 (Fig. 4E). 10% of GFP-labeled hilar interneurons showed an overlap with Parvalbumin (Fig. 4F), a marker for basket cells (12 cells out of 110; n = 4; Fig. 4F).

### Proliferative activity of DCX-GFP expressing cells in the adult dentate gyrus

The proliferative activity of GFP-expressing cells and their progression through developmental stages in the dentate gyrus was characterized using S-phase marker BrdU, which permanently labels dividing cells (Fig. 3A). At day 1, 110 out of 150 GFP+ cells (n = 3), and at 3 days 122 out of 150 cells (n = 3) had incorporated BrdU following a single injection. Most of these proliferating cells were classified as horizontal type-2 cells. In transgenic mice that received a three-day series of BrdU injections 128 out of 150 GFP+ cells (n = 3) were BrdU+ when assessed two weeks following the last injection. Further analysis revealed a few GFP/CR/BrdU+ cells (15 out of 150 cells; n = 3 (Fig. 4D) one day following BrdU, but no NeuN coexpression was detected at either time. These data indicate that DCX in transgenic mice is rapidly down regulated in more mature postmitotic neurons labeled categories E (when one strong apical dendrite is branching into the molecular layer) and F (with delicate dendritic trees branching into the granule cell layer) in a previous publication by our group [14].

### DCX-GFP expression pattern in the piriform cortex

We next studied DCX reporter gene expression in the piriform cortex. This three-layered brain region contains different types of principal neurons and interneurons with distinct morphologies and anatomical locations. The populations of neurogliaform cells and semilunar-pyramidal neurons have been previously characterized by PSA-NCAM immunoreactivity [19], [20]. Confocal images in Figure 5 reveal strong DCX-GFP expression in neurogliaform cells and semilunar-pyramidal neurons in layer II, fainter in deep/large pyramidal neurons located in layer III, and some interneurons.

**Figure 5:** Phenotypic marker expression and distribution of DCX-GFP cells in the adult piriform cortex (Bregma –0.82/2.98). (**A**) Bright and abundant GFP expression is observed in neurogliaform cells in layer II in close proximity to layer I, whereas semilunar-pyramidal neurons (arrows in layer II) and deep/large pyramidal neurons (arrowheads in layer III) show partly faint GFP signaling. (**B**) DCX-protein (in blue) is mainly expressed by neurogliaform cells that often form clusters (arrowheads) around semilunar pyramidal neurons (arrow) with only weak GFP but strong DCX-protein expression (B1–B3); the broken arrow displays a semilunar-pyramidal neuron with stronger GFP signaling, while no DCX overlap was found in morphology-wise interneuron populations (asterisk). (**C, C′**) NeuN (in blue) is expressed by all deep/large pyramidal neurons (DP) with the typical apical dendrites (small arrows), and by approximately 60% of semilunar-pyramidal neurons (SP; C1–C3). Only a few neurogliaform cells (NG), and some horizontal (H) interneurons are NeuN+. (**D–E**) Some GFP+ cells in layer II and III express the interneuron marker Parvalbumin (in blue, arrow), and Calretinin (in red, arrows), in addition to a third of neurogliaform cells that are also CR+ (E′, E1-3), asterisk marks CR+ but GFP- cells. Scale bar 150 µm.

Quantitatively, a high density of small neurogliaform cells with short and locally ramified processes was observed in close proximity to layer I (Fig. 5A). The majority of these cells were DCX+ when compared with DCX-antibody (102 out of 160 cells; n = 4; Fig. 5B), and they often form clusters surrounding principle cells with faint GFP signaling but strong native DCX-expression (Fig. 5B). Neurogliaform cells to some degree expressed the neuronal marker NeuN (38 out of 150 cells; n = 4; Fig. 5C), and also CR (31 out of 150 cells; n = 3; Fig. 5E).

Furthermore, layer II is enriched with cell bodies of semilunar-pyramidal neurons, a principal cell population and primary target of olfactory information [47]. These cells displayed partly less GFP fluorescence intensity with two apical processes extending towards layer I (Fig. 5A). Detailed phenotypic analysis revealed that one third of GFP+ semilunar-pyramidal neurons coexpressed DCX-antigen (45 out of 150 cells; n = 4; Fig. 5B), whereas a greater percentage expressed NeuN (94 out of 150 cells; n = 4; Fig. 5C).

Layer III is formed by deep/large pyramidal neurons with likewise faint GFP-expression in soma and cell body but clearly recognizable apical dendrites extending towards layer I (Fig. 5C). No overlap with DCX-protein was observed (150 cells analyzed in n = 3 animals). Yet all GFP+ deep/large pyramidal neurons expressed NeuN (150 cells analyzed in n = 4 animals; Fig. 5C).

In addition, small populations of interneurons that are not neurogliaform cells were characterized by coexpression of GFP and CR or Parvalbumin, and have been observed with fainter GFP signaling in layer II and III (Fig. 5D, E). These cells have been earlier described as bitufted B, and multipolar M cells, respectively [28]. Based on morphology, a very few horizontal (H) NeuN+ interneurons could be identified in layer I (Fig. 5C).

We did not detect any co-labeling for glial markers in GFP+ cells.

Next, we investigated the proliferative activity of GFP+ cells in the adult piriform cortex with the help of BrdU injected at different time points. None of the cells in the identified populations of GFP+ cells was BrdU+ either at one, three days or two weeks after the BrdU injection.

The few proliferating BrdU+ cells found in the piriform cortex typically expressed the proteoglycan NG2, characteristic of the proliferating cell populations outside neurogenic regions, or S100β.

### Membrane properties of DCX-GFP expressing cells in the adult dentate gyrus

To determine the electrophysiological properties of GFP-expressing newly generated cells in the adult DG, cells were voltage-clamped and dye-filled. Two populations of GFP+ cells were distinguished based on their fluorescent intensities (weak and bright cells; Fig. 6A). Membrane properties are listed in Table 1. Weak cells had a significantly higher negative membrane potential (−69±1 mV) and a lower membrane resistance (Rm) relative to bright cells. The membrane resistance of Rm = 4.0±0.4 for weak cells is similar to previously reported properties of newly generated granule cells [43]. Furthermore, depolarizing voltage steps from a holding potential of −70 mV to −30 mV elicited relatively low Na^+^ currents in weak cells (71±8 pA) typical of immature neurons (Fig. 6B). Thirty to 40% of both cell populations exhibited a clear single action potential under current clamp configuration (80 pA current injection for 200 ms, Fig. 6C). Nevertheless, the majority of GFP+ cells in the adult DG are immature and non-excitable. No spontaneous postsynaptic currents were detected (Fig. 6D).

**Figure 6:** Physiological properties of DCX-GFP-expressing cells in the adult piriform cortex in comparison to the DG. GFP+ cells (green) from adult mouse brain slices were patch-clamped with a glass pipette and filled with 10 µg/ml Alexa Fluor 594 (red). (**A**) Images of a neurogliaform cell, a semilunar-pyramidal neuron, and a large pyramidal neuron in the piriform cortex; bright and weak cells in the dentate gyrus. The patched cell is enlarged shown in a small box above. Cortical layers are marked as I, II, and III. (**B**) Large Na^+^ currents were detected in deep pyramidal neurons, whereas neurogliaform cells and dentate newly born neurons had small Na^+^ currents. (**C**) Single and multiple action potentials were elicited by 200 ms current injection of 30 and 80 pA in the piriform cortex and dentate gyrus, respectively. (**D**) Spontaneous current were detected in a proportion of semilunar-pyramidal neurons and large pyramidal neurons of the piriform cortex but not in newly generated cells of the dentate gyrus; NG, neurogliaform cells, SP, semilunar-pyramidal neurons, DP, large/deep pyramidal neurons.

**Table 1:** Electrophysiological properties of DCX-GFP-positive cells in the dentate gyrus (** p<0.01).

	Bright cells	Weak cells
N	18	27
Membrane Potential Vm (mV)	−62±1	−69±1**
Membrane Resistance Rm (GΩ)	1.3±0.3	4.0±0.4**
Maximum Na^+^ current (pA)	126±37	71±8
Cells with elicited single action potentials (%)	8/18 (44%)	9/27 (33%)

### DCX-GFP-expressing cells in the piriform cortex exhibit electrophysiological properties of mature cells

The populations of GFP+ neurogliaform cells, semilunar-pyramidal neurons, and deep/large pyramidal neurons were detected and distinguished by a characteristic morphology and fluorescent intensity (Fig. 6A). Membrane properties of each cell type are listed in Table 2. While bright neurogliaform cells in layer II showed similar features as detected for newly generated granule cells such as low Na^+^ currents (220±49 pA), GFP+ cells described as semilunar-pyramidal neurons and deep/large pyramidal neurons revealed significant differences with large Na^+^ currents (pA = 1408±383 and 2106±405, respectively; Fig. 6B). Under current clamp (30 pA current injection for 200 ms) half of neurogliaform cells in layer II elicited single action potentials, whereas both single and multiple action potentials were found in 86% (12 out of 14 cells) of semilunar-pyramidal neurons and in 100% (7 out of 7 cells) of deep/large pyramidal neurons (Fig. 6C). Both cell populations also showed spontaneous postsynaptic currents (4 out of 11 cells −36% and 3 out of 7 cells −43%, respectively; Fig. 6D). Together, the majority of GFP+ cells in the piriform cortex are mature neurons with large Na^+^ currents and multiple action potentials.

**Table 2:** Electrophysiological properties of DCX-GFP-positive cells in the piriform cortex (** p<0.01; neurogliaform cells as control).

	Neurogliaformcells	Semilunar-pyramidal neurons	Large pyramidal neurons
N	10	14	7
Membrane Potential Vm (mV)	−67.0±1.3	−66.7±0.9	−66.0±1.4
Membrane Resistance Rm (GΩ)	2.8±0.5	2.7±0.7	2.3±0.9
Maximum Na^+^ current (pA)	220±49	1408±383 **	2106±405**
Cells with elicited action potentials (%)	5/10 (50%)	12/14 (86%)	7/7 (100%)
Cells with spontaneous current (%)	0/10 (0%)	4/11 (36%)	3/7 (43%)

## Discussion

In the present study we have shown that DCX expression in the piriform cortex is not associated with adult neurogenesis as it is in the hippocampus but possibly with other types of plasticity. The strong DCX expression in the piriform cortex and the intriguing location between two neurogenic regions (Fig. 1) had stimulated particular interest in the DCX+ population of the piriform cortex. In some cases, DCX expression alone has been taken as indication of adult neurogenesis [32], [48] but this step is problematic. These as well as other related reports (see introduction) had not taken functional characterization into account. We thus took advantage of a DCX-reporter mouse and electrophysiological analyses to describe the DCX-positive cells of the piriform cortex. We made efforts to compare the DCX+ cells of the piriform cortex to those of the dentate gyrus. This is the first study to investigate electrophysiological properties of DCX+ cells outside the canonical neurogenic regions.

Doublecortin is clearly an interesting marker molecule to study neuronal differentiation of newly generated cells in neurogenic regions of the adult brain. In the course of adult hippocampal neurogenesis transient DCX expression characterizes migration and links the neuronal precursor cell stage with a postmitotic immature stage [4], [14]. The functional role of DCX has as yet not been thoroughly investigated but appears to be linked to microtubule stability [49]. DCX is expressed in migratory cells and has been discovered because of its mutation that causes disturbed cortical lamination in humans. DCX plays a similar role for hippocampal lamination [11].

Our data demonstrate that GFP expression in the hippocampus reflected the known expressing pattern of DCX expression cell stages in the SGZ (type 2b, 3 and early immature postmitotic neurons [45]) but emphasizes the early high proliferative stages. Furthermore, GFP expression is rather weak in the processes of DCX-GFP+ cells. This suggests that the DCX promoter is down regulated in postmitotic cells that are still DCX-protein-immunoreactive.

In the piriform cortex, different neuronal phenotypes were still GFP+ in the absence of DCX-antigen-labeling and co-expressed NeuN. Our findings confirm three classes of neuronal cell types that could be detected with the reporter mouse. Whereas neurogliaform cells mostly expressed DCX protein and shared physiological properties with newly generated neurons in the DG, semilunar-pyramidal neurons and deep/large pyramidal neurons mainly expressed the mature neuronal marker NeuN, and spontaneous postsynaptic currents and large Na^+^ currents were detected. In addition to large Na^+^ currents, the majority of GFP+ cells in layer II and III elicited multiple action potentials under current clamp configuration. In addition, some CR+ and Parvalbumin+ interneurons with weak GFP expression were found.

Newly generated granule cells in the adult DG with DCX expression show physiological properties such as low Na^+^ currents and a strong negative resting potential and feature enhanced excitability and increased levels of synaptic plasticity, e.g. a lower threshold for LTP [43], [50], [51], [52].

The piriform cortex functions as relay station for processing olfactory information and continuously receives new input via afferent excitatory fibers that predominantly synapse with semilunar-pyramidal neurons in layer I [27], [47], [53]. Neurogliaform cells characterized as an interneuron population may be also target by extrinsic afferent fibers (as previously described for horizontal interneurons in layer 1 by [28]) and mediate feed-forward inhibition onto principal cells. In our study, neurogliaform cells form clusters around principal cells and share similar features to newly generated granule cells. Piriform cortex interneurons can also participate in long-term potentiation (LTP), where GABAergic inhibition in principal dendrites needs to be blocked so that associative LTP can be induced [54]. Here, strong DCX-GFP expression features enhanced synaptic plasticity that is necessary to adapt to environmental changes and to process olfactory information. Although a few CR+ and Parvalbumin+ cells were found playing a role in feedback inhibition, GFP signaling was only weak, and cells do not constitute the major DCX-GFP expressing population.

Throughout the brain, NG2-positive cells faintly expressing DCX have been reported [55], [56], [57] and we have found these cells also in the dentate gyrus. We did not detect them in the piriform cortex proper. It is thus not clear, whether any lineage-relationship exists here. Generally, NG2 cells represent a new class of glial cells (for review see [58], [59], [60]). They were termed complex glial cells, polydendrocytes or simply NG2 cells. In the hippocampus, these cells are also weakly GFAP-positive [61].

We found that DCX-expressing cells in the piriform cortex are strictly postmitotic with no overlap of BrdU at one or three days, or two weeks after BrdU injection. Based on morphology we also could not identify migrating neurons in layers II or III of the adult piriform cortex. This does not strictly preclude that DCX-expressing cells might be generated from a DCX-negative population outside the hippocampus with a maturation time of more than two weeks before the onset of DCX expression. Potentially, genetic lineage tracing or different labeling protocols might reveal such cases, especially if the precursor cells only occasionally divide. Long-term labeling with BrdU, however, is not without problems [62], [63]. It does speak against the presence of DCX-positive, proliferative intermediate progenitor cells (type-2b in the dentate gyrus) and “neuroblasts” (type-3) in the piriform cortex.

DCX-GFP transgenic reporter mouse is a powerful tool to visualize different cell types in the adult brain *in vivo*, and even more to analyze their physiological properties. DCX-GFP expression is abundant in areas of continuous neurogenesis, but was also detected in the non-neurogenic piriform cortex. Our present data support the idea that DCX-expressing cells do not constitute a homogeneous population in the adult brain. However, DCX signifies transient neuronal lineage commitment together with migration and neural structural plasticity in the adult hippocampal niche, and indicates synaptic plasticity in the adult piriform cortex layer II, that is necessary for rapid adaptation to environmental changes. Our data indicates that while DCX represents a dividing progenitor population in the neurogenic niche of the hippocampus it also labels a non-dividing neuron with immature traits in the non-neurogenic niche of the piriform cortex.
